This article has been retracted.

# Prognostic Utility of Coronary Computed Tomographic Angiography: A 5-Year Follow-Up in Type 2 Diabetes Patients with Suspected Coronary Artery Disease

**DOI:** 10.1155/2014/103459

**Published:** 2014-03-09

**Authors:** Daliang Liu, Huijuan Jia, Yucun Fu, Wen He, Daqing Ma

**Affiliations:** ^1^Department of Radiology, Beijing Friendship Hospital, Capital Medical University, 95 Yongan Road, Xicheng District, Beijing 100050, China; ^2^Department of Radiology, Liaocheng People's Hospital, 67 West-Dongchang Road, Liaocheng, Shandong 252000, China

## Abstract

*Objectives.* To analyze the predictive value of coronary computed tomography angiography on acute coronary artery events in patients with type 2 diabetes. *Methods.* Coronary computed tomography angiography was performed in 250 type 2 diabetic patients. After a follow-up for 5 years, 145 patients were excluded as they did not have any coronary events. The remaining 95 patients were divided into study group and control group. According to their density and shape, the coronary artery plaques were classified into 3 types and 4 types, respectively. *Results.* There is no statistically significant difference in the degree of stenosis between two groups. The proportion of calcified plaques in the study group was lower than in the control group. The proportion of mixed-calcified plaques in the study group was higher than in the other. Type III plaques have a 76.2% sensitivity and negative predictive value was 64.5% for acute coronary events; type IV plaques have a sensitivity of 52.6% and positive predictive value of 63% for chronic coronary events. *Conclusions.* CCTA may be used as a non-invasive modality for evaluating and predicting vulnerable coronary atherosclerosis plaques in patients with type 2 diabetes.

## 1. Introduction

Type 2 diabetes mellitus (T2DM) is a major risk factor for cardiovascular disease and is associated with significant cardiovascular morbidity and mortality [1]. Patients with T2DM have increased risk of major adverse cardiac events (MACE) [1]. Acute coronary events are often caused by the rupture of unstable coronary atherosclerotic plaques and coronary stenosis [2, 3]. Therefore, assessment of atherosclerotic plaque morphology and pathological features has become an important part of clinical investigation of coronary artery disease [4]. Multidetector coronary computed tomography angiography (CCTA) has been increasingly used in the evaluation of the coronary arteries [5]. In an acute setting, CCTA is associated with 95% sensitivity and 90% specificity in diagnosing non-ST-elevation myocardial infarction (NSTEMI) and unstable angina pectoris [6]. The ability to detect not only coronary stenosis but also the nonobstructive coronary atherosclerotic plaques in a noninvasive fashion makes CCTA imaging a potentially valuable tool for risk stratification. In recent years, CCTA has been used to predict the prognosis or cardiac events in patients with suspected coronary artery disease [7–14]. However, there has been limited information on the predictive value of CCTA on the acute coronary events in patients with T2DM.

The purpose of this study is to investigate the CCTA characteristics of the coronary plaques in patients with T2DM. The sensitivity and specificity of CCTA in predicting the acute coronary events in these patients are also evaluated.

## 2. Subjects and Methods

### 2.1. Study Population

The study was approved by the Institutional Ethics Committee of our hospitals, and written informed consent was obtained from all participants. From February 2007 to November 2008, 318 consecutive patients with T2DM were referred to our department for coronary CTA because of nonspecific chest pain, exertional dyspnea, or ST-T depression or flattening on electrocardiogram (ECG). Patients who had a previous coronary balloon angioplasty, stenting, or coronary artery bypass grafting were excluded. Other exclusion criteria were (a) heart rate above 90 beats/min or with atrial fibrillation or other arrhythmias; (b) renal dysfunction (serum creatinine ≥ 120 mmol/L); (c) other chronic illnesses, such as severe respiratory insufficiency, hyperthyroidism; (d) inability to give a written consent. In the end, 250 patients were recruited to this study and 68 were excluded. The reasons for exclusion are listed in Figure 1.

### 2.2. CCTA Protocol

The first 85 patients were scanned by Philips Brilliance 64-detector CT (Philips Medical Systems, Eindhoven, The Netherlands). Prior to the scans, beta-blocker was administered in patients whose heart beat was ≥70/min, and nitroglycerine (0.3 mg sublingually) was used in all patients 15 minutes before the scans. Retrospective ECG-gated helical CCTA was performed in 64-detector CT. The scan parameters were 64 × 0.625 mm collimation, 120 kV tube voltage, 400–600 mAs tube current, 0.42 s rotation time, and 0.2 pitch. Data acquisition was completed within 4.1–5.9 sec with radiation dose of 13.9–16.8 mSv (median, 15.1 mSv). In the remaining 65 patients, prospective ECG-gated scan was performed in 128-detector CT and heart rate was restricted within 60–70 beats/min. The scan parameters were 120 kV tube voltage, 200 mAs tube current, collimation 128 × 0.625, 0.18–0.27 sec rotation time, and 0.2 pitch. Scanning was completed within 3.9–6.8 sec with radiation dose of 3.16–4.14 mSv (median, 3.6 mSv).

A 50–60 mL (dependent on body mass index) bolus of iodinated contrast agent (iopamidol, 370 mg of iodine/mL; Bracco Sine Pharmaceutical Corp. Ltd., Shanghai, China) was injected into the antecubital vein at a flow rate of 4-5 mL/sec. The scanning range was from the tracheal bifurcation to 10 mm below the inferior cardiac apex. The best quality images were chosen for evaluation and other phases or ECG-editing was performed if needed. All initial data sets were transferred to a postprocessing workstation (Brilliance-workshop, Philips Medical Systems, Eindhoven, The Netherlands) for image analysis. Alternative image reconstruction methods for evaluation of coronary artery and plaques included maximum intensity projection, multiplanar reconstruction, curvature plane reconstruction, and volume rendering.

### 2.3. Stenosis and Plaque Analysis

Two cardiovascular radiologists analyzed the images independently. Both observers were blinded to the medical histories, clinical diagnoses, and results of other investigations for all patients. In case of disagreement, the features of plaque and stenosis evaluations were reevaluated for the consensus judgment.

Subsequently the type of plaque was determined: noncalcified, calcified, or mixed [15]. Noncalcified plaques are plaques with a lower density compared with the contrast-enhanced lumen; calcified plaques are plaques with a higher density; and mixed plaques are plaques with soft and calcified elements within a single plaque. The measure was performed in axial and MPR images and 4 points were chosen randomly. ROI > 1.0 mm^2^ (at least 3 contiguous pixels, area 1.03 mm^2^) and the smallest CT value were defined as the value of plaques (Figures 2 and 3). The coronary artery plaques were classified into 4 types [16, 17]: type I, concentric lesions; type II, eccentric lesions with a wide base but smooth margin; type III eccentric lesions with a narrow base and rough surface; type IV, long segment of irregular lesions.

Number of diseased coronary vessels and segments, number and types of plaques, and grading of stenosis caused by plaques were evaluated. Coronary arteries were divided into 15 segment models of the American Heart Association [18]. The involved vessels were classified as single, double, and triple vessels. The degree of stenosis was defined as the percentage of stenosis and adjacent normal vessel lumen: normal or mild (<50%), moderate (50%–75%), and severe (≥75%) stenosis [19].

### 2.4. Follow-Up

The follow-up was conducted by structured telephone interviews with patients or the relatives who knew the patients' conditions. The follow-up questionnaires included the general health of the patients, use of medications, cardiovascular events including hospital admissions, coronary artery angiography or stenting, or coronary artery bypass grafting. The interviews were conducted every 6 months for 5 years.

The acute coronary events were defined as acute coronary syndrome (ST-elevation or Non-ST elevation myocardial infarction, or unstable angina) or sudden cardiac death (study group). Patients with stable angina, or with angiographically identified coronary artery stenosis requiring elective coronary stenting or bypass grafting 6 months after CCTA, were considered as having chronic coronary events [14] (control group).

### 2.5. Statistical Analysis

Data are expressed as means ± standard deviation (SD). Chi-square test was used to compare the categorical data between the study and control groups. *P* value of <0.05 was considered statistically significant. All statistical analyses were performed using the SPSS statistical package (version 11.5 for Windows, SPSS Inc., Chicago, IL, USA).

## 3. Results

### 3.1. General Findings

A total of 318 patients were recruited in this study but 150 completed the follow-up (Figure 1). The baseline characteristics of these patients are summarized in Table 1.

During the follow-up period, acute coronary events occurred in 28 (18.7%) patients, including acute myocardial infarction in 8 (5.3%); unstable angina in 19 (12.7%); and sudden death in 1 (0.7%). Within the first 6 months of the follow-up, 15 patients with the acute coronary events had coronary stenting and 8 received coronary bypass grafting. Chronic coronary events occurred in 67 (44.7%) patients, including stable angina pectoris in 58, elective coronary stenting in 7, and elective coronary bypass grafting in 2. The remaining 55 (36.7%) patients were asymptomatic and free of coronary events during the follow-up.

### 3.2. Coronary Artery Plaques on CCTA Images

A total of 420 segments were analyzed in study group and 1005 segments were analyzed in control group (Table 2). Triple-vessel diseases were identified in 67.8% of the study group and in 68.6% of the control group (*P* = 0.380). Moderate-to-severe degree of coronary stenosis was found in 89.8% of the study group and in 88% of the control group (*P* = 0.380).

The numbers and characteristics of coronary plaques in the study and control groups are shown in Table 3. In the study group, there were 236 noncalcified, 315 mixed, and 87 calcified plaques. In the control group, the noncalcified, mixed, and calcified plaques were 48, 596, and 843, respectively. The proportion of calcified plaques in the study group was lower than in the control group (13.6% versus 53.2%, *P* < 0.01). The proportion of noncalcified plaques in the study group was higher than in the control group (37% versus 9.3%, *P* < 0.001).

### 3.3. Plaque Morphology and Acute Coronary Events

The numbers of different plaque types founded on CCTA images are listed in Table 4. In the study group, there was no statistically significant difference in the plaque types between patients with moderate or severe coronary stenosis (*P* = 0.349). In the control group, however, there was a statistically significant difference in the plaque types among different grades of stenosis in the control group (*P* < 0.001).

As shown in Table 4, there was no statistically significant difference in the proportion of type I plaques between the study and control groups (*P* > 0.05). However, the proportion of type III plaques in the study group was higher than in the control group, whereas the proportion of type II and IV plaques was lower (*P* < 0.01).

Using type III plaques to predict acute coronary events, the sensitivity and specificity were 76.2% and 63.8%, respectively.

## 4. Discussion

The main findings of the present study are as follows: (a) the proportion of noncalcified and type III plaques in patients with acute coronary events was higher than in patients with stable angina; (b) the proportion of calcified plaques in patients with stable angina was higher than in patients with acute coronary events; (c) the sensitivity and specificity of type III plaques in predicting acute coronary events were 63.8% and 76.2%, respectively. The sensitivity and specificity of type II and IV plaques in predicting chronic coronary events were 91.5% and 79%, respectively. These findings indicated that noninvasive CCTA may be used to evaluate the unstable plaques that are prone to cause ACS in patients with T2DM.

Previous studies have found that many coronary lesions in patients with coronary heart disease were nonobstructive, and the vessel with mild-to-moderate stenosis was responsible for cardiac events [20, 21]. The vulnerability of the intracoronary lesions is a key factor for ACS in these patients with mild-to-moderate stenosis [20, 21]. Acute coronary syndrome was often caused by rupture of coronary artery atherosclerosis plaques rather than lumen stenosis [22]. Therefore, early detection of vulnerable or unsteady plaques is important in guiding prevention and treatment of acute cardiac events. Noncalcified plaques were unsteady and were commonly seen in patients with acute coronary syndromes [23, 24]. Inconsistent with the previous reports, our study showed that there was little difference in the stenosis severity between patients with acute and chronic coronary events. On the other hand, the types of the coronary plaques on CCTA seem to be related to the coronary events. We also found that, in patients with acute coronary syndromes, there were more noncalcified plaques and fewer calcified plaques than in patients with stable angina. These results suggest that, in patients with T2DM, analysis of the stenosis severity alone on CCTA is probably insufficient. Evaluation of the plaque morphology and vulnerability on CCTA seems to offer additional information on the future risk of acute coronary events.

The reliability of CCTA in assessing coronary plaque stability has been under investigation in recent years [25–28]. The study of Otaki et al. [28] showed the prognostic information of CCTA enhances risk stratification and may improve medical therapy and/or behavioral changes that may enhance event-free survival. An earlier study by Motoyama et al. [29] demonstrated that CCTA can be used to accurately assess plaque composition by measuring the CT value of the plaque on thin-CT images. Falk et al. [30] reported that eccentric lesion was an index of unsteady plaques. The lipid core was in the inner lining of the coronary lumen and was prone to rupture under the impact of blood flow. The ruptured plaques will absorb platelets, leading to new clots formation and obstruction of coronary flow and causing acute coronary syndrome or sudden death [31]. In the present study, we have divided the coronary plaques into 4 types [16, 17]. The type III plaques, those with an eccentric centre and rough surfaces, appear to be related to acute coronary events. The predictive sensitivity and specificity of type III plaques were 63.8% and 76.2%, respectively, for acute coronary events. On the other hand, eccentric lesions with a wide base but smooth margin (type II plaques) and long segment of irregular lesions (type IV plaques) represent relatively stable plaques and have 91.5% sensitivity and 79% specificity in predicting chronic coronary events.

Achenbach and Raggi [32] thought that the actual clinical utility of coronary CTA for risk stratification purposes is very uncertain, especially when considering extending the currently available findings to a “screening” situation. Many trials [33–36] which demonstrated a prognostic value of coronary CTA were all retrospective analyses of individuals in whom CT was performed for a clinical reason, so most likely the populations mainly consisted of symptomatic patients. Because of the low overall event rate, predicting acute coronary syndromes in asymptomatic individuals is substantially more difficult. So ADA 2013 guideline pointed that, for asymptomatic patients, it is not recommended for routine screening for CAD, because this screening does not make sense to improve the outcomes as long as appropriate treatment for CAD risks can be achieved [37].

But similar to the detection and quantification of coronary calcium, one would expect that the detection and further characterization of noncalcified plaque should provide prognostic information concerning the occurrence of future acute coronary syndromes. Ostrom et al. [33] demonstrated that the presence of nonobstructive plaque in all three coronary arteries was associated with increased mortality (risk ratio 1.77 when compared with individuals without any detectable plaque). Hausleiter et al. [38] proposed that the burden of angiographic disease detected by CTA provides both independent and incremental value in predicting all-cause mortality in symptomatic patients independent of age, gender, conventional risk factors, and CAC. So we should do more research to find unstable plaque or criminal vessels.

A further concern is the fact that CCTA, as opposed to coronary calcium, requires the injection of contrast agent and is usually associated with substantially higher radiation exposure than calcium scans. Average effective doses for CCTA are 12 mSv, but they can easily reach 20 mSv or more unless special measures to minimize the dose are implemented [33, 39]. Recently, numerous approaches to reduce the dose of CCTA have been proposed and evaluated, and estimated effective doses, 3 mSv [40–43] in selected cases even 1 mSv [44], can be achieved.

A potential limitation of the present study on the first 85 patients is that, in the earlier part of our study, retrospective ECG-gated helical CCTA was performed using 64-detector CT. In the remaining 65 patients, prospective ECG-gated scan was performed using 128-detector CT. The imaging quality of 128-detector CCTA is generally superior to 64-detector CCTA and the dose of radiation is also lower [5, 31]. Indeed, we excluded 7 patients from the study due to poor imaging quality. All of these excluded patients were scanned with 64-detecor CCTA. Another limitation is the small number of cases. So we need do more research to discover how predictive the CCTA is versus traditional risk assessment.

## 5. Conclusions

CCTA is a noninvasive modality to measure the severity of coronary stenosis and to assess the morphology of coronary plaques and provides potential prognostic information in T2DM patients with suspected CAD. These data suggest morphology analysis on CCTA may add value to coronary risk stratification in patients with T2DM although more studies are needed. These results may improve the risk stratification in patients evaluated by CCTA and provide strategies for the individualized prevention programs.

## Figures and Tables

**Figure 1:** Flow chart of the study participants.

**Figure 2:** A 51-year-old female with an 8-year history of type 2 diabetes. Soft plaques were identified in the left descending coronary artery with an eccentric and unsmooth surface (black arrow). CT value was 28 Hu.

**Figure 3:** A 57-year-old female with an 11-year history of type 2 diabetes. Mixed plaque was showed in LAD with eccentric lesions with a narrow base and rough surface (black arrow).

**Table 1:** Baseline characteristics.

Characteristic	Study group (*n* = 28)	Control group (*n* = 67)	*P* value
Age (years)	64.7 ± 14.6	63.6 ± 15.3	NS
Male sex	16 (57.1)	29 (43.3)	NS
BMI, kg/m^2 ^	25.8 ± 3.54	25.3 ± 1.49	NS
Other cardiovascular risk factors			
Hypertension	17 (60.7)	42 (62.7)	NS
Hypercholesterolemia	13 (46.4)	32 (47.8)	NS
Smoking	15 (53.6)	34 (50.7)	NS
Family history of CHD	9 (32.1)	21 (31.3)	NS
Clinical presentation			
Abnormal electrocardiogram	24 (85.7)	46 (68.7)	NS
Atypical angina	8 (28.6)	27 (40.3)	NS
Nonspecific chest pain	17 (60.7)	38 (56.7)	NS
Dyspnea	18 (64.3)	45 (67.2)	NS
Diabetes treatment			
Oral agents	2 (7.1)	12 (17.9)	NS
Oral agents plus insulin	26 (92.8)	55 (82.8)	NS

Note: data are numbers of patients except where indicated otherwise. Numbers in parentheses are percentages. BMI: body mass index.

**Table 2:** Comparison of coronary lesions and degree of coronary stenosis between groups.

	Study group (*n* = 28)	Control group (*n* = 67)	*P* values
Vessels involved			
Single	4 (14.4%)	8 (12%)	NS
Double	5 (17.8%)	13 (19.4%)	NS
Triple	19 (67.8%)	46 (68.6%)	NS
Stenosis grade			
<50%	43 (10.2%)	121 (12.0%)	NS
50%–75%	263 (62.6%)	641 (63.8%)	NS
≥75%	114 (27.2%)	243 (24.2%)	NS

NS: no significant difference.

**Table 3:** The comparison of plaques number and characteristic between study and control groups.

Plaque characteristics	Study group (plaques = 638)	Control group (plaques = 1586)	*P* values
Noncalcified	236 (37%)	148 (9.3%)	<0.001
Mixed	315 (49.4%)	595 (37.5%)	<0.001
Calcified	87 (13.6%)	843 (53.2%)	<0.001

**Table 4:** Comparison of plaque morphology between study and control groups.

Plaque morphology	Study group (*n* = 638 plaques)	Control group (*n* = 1586 plaques)	*P* value
Type I	38 (6%)	89 (5.6%)	0.825
Type II	65 (10.2%)	637 (42.2%)	<0.001
Type III	486 (76.2%)	276 (17.4%)	<0.001
Type IV	49 (7.6%)	584 (36.8%)	<0.001
